# Lung Disease Classification in CXR Images Using Hybrid Inception-ResNet-v2 Model and Edge Computing

**DOI:** 10.1155/2022/9036457

**Published:** 2022-03-30

**Authors:** Chandra Mani Sharma, Lakshay Goyal, Vijayaraghavan M. Chariar, Navel Sharma

**Affiliations:** ^1^Indian Institute of Technology Delhi, Delhi, India; ^2^Veritas Technologies LLC, Pune, India; ^3^Academic City College, Accra, Ghana

## Abstract

Chest X-ray (CXR) imaging is one of the most widely used and economical tests to diagnose a wide range of diseases. However, even for expert radiologists, it is a challenge to accurately diagnose diseases from CXR samples. Furthermore, there remains an acute shortage of trained radiologists worldwide. In the present study, a range of machine learning (ML), deep learning (DL), and transfer learning (TL) approaches have been evaluated to classify diseases in an openly available CXR image dataset. A combination of the synthetic minority over-sampling technique (SMOTE) and weighted class balancing is used to alleviate the effects of class imbalance. A hybrid Inception-ResNet-v2 transfer learning model coupled with data augmentation and image enhancement gives the best accuracy. The model is deployed in an edge environment using Amazon IoT Core to automate the task of disease detection in CXR images with three categories, namely pneumonia, COVID-19, and normal. Comparative analysis has been given in various metrics such as precision, recall, accuracy, AUC-ROC score, etc. The proposed technique gives an average accuracy of 98.66%. The accuracies of other TL models, namely SqueezeNet, VGG19, ResNet50, and MobileNetV2 are 97.33%, 91.66%, 90.33%, and 76.00%, respectively. Further, a DL model, trained from scratch, gives an accuracy of 92.43%. Two feature-based ML classification techniques, namely support vector machine with local binary pattern (SVM + LBP) and decision tree with histogram of oriented gradients (DT + HOG) yield an accuracy of 87.98% and 86.87%, respectively.

## 1. Introduction

Machine learning is very useful in healthcare informatics. It has applications in disease diagnosis, classification, and prognosis. Computed tomography (CT) scan and CXR imaging are two very commonly used diagnostic techniques used for the detection of lung diseases [1–4]. The detection of lung diseases has gained a lot of popularity due to the prevailing COVID-19 spread. Much work has been done in the recent past. However, there is a demand to utilize the power of edge computing for disease detection. Most of the systems for lung disease classification are either stand-alone or cloud-based. We used the CXR dataset compiled by Rahman [5, 6], which is freely available for research purposes [5]. It was first used to detect and classify COVID-19 and viral pneumonia [7]. Deep neural network-based models have been successful in learning the discriminative features in image-based disease classification tasks such as tuberculosis detection [1] and lung disease classification [3] in radiographs [1] and lung nodule classification in CT scans [2, 4].

Furthermore, CXR can be used as a tool for diagnosing a number of diseases and complications, such as thoracic diseases, fractures, tooth decay, infections, osteoporosis, enlarged hearts, blocked blood vessels, etc [2, 4, 7]. At present, the world is grappling with COVID-19, with Omicron being the most recent variant of concern. There are different diagnostic tests available to screen and diagnose the disease. Owing to the easy availability of chest X-ray imaging facilities and cost-effectiveness, it is chosen as one of the preferred methods for COVID-19 detection as well [6, 7]. Radiology expertise is required in order to distinguish COVID-19 from other diseases. However, there is an acute shortage of trained radiologists. X-ray imaging is a very common diagnostic test performed to diagnose upper respiratory diseases such as pneumonia, COVID-19, fluid in the lungs, etc. With the advent of improved hardware and software capabilities, it is now possible to train machine learning classifiers on large datasets with human-comparable accuracy.

In contrast with CT scan, CXR may be advantageous for the following reasons:

- The limited specificity of CT scanning might make it difficult to discover non-COVID-19 cases. Furthermore, the rays from CT scanners might pose complications for individuals who need frequent CT scans throughout their illness.
- Color information, with its variables such as color composition, light beams, and reflections, causes various issues.
- X-ray imaging is far more common and less expensive than traditional diagnostic examinations.
- X-rays have several advantages over CT scans, including being faster, safer, easier, and less damaging.
- Problems include the possibility of disease transmission when utilizing a CT scan scanner, as well as the technology's expensive cost, which can generate major issues for patients and healthcare systems.

Edge computing brings compute power closer to the source. It can be advantageous for deploying disease detection systems in many ways, such as low latency, high speed, and can achieve economies of scale with the help of edge devices [8]. A review of previous works to deploy machine learning and deep learning models for COVID-19 detection and mitigation in edge environments [8, 9] inspired the current study.

A great deal of research has been done on the detection of COVID-19 in CXR images. Researchers have attempted to resolve the problem in a variety of ways, resulting in the development of new classifiers, datasets, preprocessing techniques, and performance metrics [2–4, 7]. While deep networks have the advantage of training models from scratch, they suffer from overfitting on small datasets. Therefore, transfer learning-based models are very popular for COVID-19 detection [10–12]. The development of end-to-end integrated applications based on edge computing, on the other hand, has received relatively little attention.

We employ a hybrid strategy of class balancing in this case, combining SMOTE and weighted class balancing. Additionally, the effect of data augmentation and image enhancement has been evaluated in order to determine the most appropriate method for use in an edge computing environment. In this study, we evaluate a number of approaches for COVID-19 detection and propose an edge computing framework for classifying lung diseases, including COVID-19, from CXR images, which is based on the results of the evaluation.

## 2. Literature Survey of the Related Work

X-ray images have many other challenges, such as complicated backgrounds and the presence of more than one potential abnormality, making the clinical analysis of X-ray images a very sophisticated task [13]. Therefore, it requires the manual annotation of experts (radiologists). The automatic analysis of X-ray images is becoming an important tool for clinical diagnosis. With the recent successes of deep neural networks in image classification, it is being widely used for X-ray image classification tasks [13–19]. Several diseases, including thoracic infections [13], COVID-19 [14, 15, 17, 19], lung abnormalities [16], etc., can be classified using deep learning on chest X-ray images. Hussain et al. [15] proposed a deep learning model, called CoroNet, for COVID-19 detection. A deep learning framework was proposed to detect lung abnormalities in CXR and CT scan images [16]. The deep learning model, proposed by Albahli et al. [17], achieved 87% accuracy using GAN-based synthetic data and presented comparable results with other techniques. Lung segmentation is another important task in CXR disease detection. It is particularly useful in establishing the severity analysis of tuberculosis [18]. A DeTraC deep convolutional neural network architecture was described by Abbas et al. [19].

Due to the hierarchical pattern exhibited by the disease [20], hierarchical classification can be useful in the detection of pneumonia. Traditional machine learning approaches like support vector machines (SVMs), k-nearest neighbour (KNN), decision tree classifiers, etc., can also be used in CXR disease classification. However, they rely on the feature extraction mechanism. Convolutional neural networks (ConvNets) can also be used as a mechanism for feature extraction. Toğaçar et al. [21] used a mRMR feature selection mechanism and compared the performance of traditional machine learning models for the detection of pneumonia. Khatri et al. [22] used earth mover's distance (EMD) to compare pneumonia CXR images. Teixeira et al. [23] used lung segmentation to assess and explain COVID-19. Multimodal approaches may aid in the better understanding and explanation of diseases in the CXR [24, 25].

Automated disease classification in X-ray images is challenging due to the unavailability of large amounts of annotated data and the efficient machine learning algorithms to learn the discriminative features from them [25]. Multiple streams and modalities of data can be used to improve the accuracy of disease prediction. The text data from X-ray diagnostic images were combined with annotated image data to train the thorax disease classifier [25]. Unlike the usual approach of directly classifying diseases, a deep disentangled generative model can be used to create residual maps for abnormal diseases along with normal images [26]. This approach helps disentangle the abnormal and normal parts of a chest X-ray. Semi-supervised generative models can be effectively used in CXR disease classification [26, 27].

There remains the possibility of simultaneous co-occurrence of more than one disease. In such a scenario, single-label classification may not work, whereas multi-label classification can solve this problem. Albahli et al. [28] proposed a CNN-based deep learning approach for multi-label classification of CXR. Further, Baltruschat et al. [29] compared several deep learning-based methods for multi-label chest X-ray classification. Pathology datasets generally contain class imbalances. It presents a risk for the trained classifier to be biased towards the majority class. Proper class balancing measures can help improve the classifier performance both in supervised and semi-supervised tests [30]. López-Cabrera et al. [31] discussed the limitations of existing machine learning-based approaches for COVID-19 detection. Tsiknakis et al. [32] proposed a framework for artificial intelligence-based interpretable COVID-19 screening using CXR images.

Edge computing has been used in many healthcare applications [33], including disease classification. Furthermore, it has applications in COVID-19 pandemic management [34–36], such as an IoT-based city lockdown system [34], social distancing management [35], and real-time mask identification [36]. However, there is very little work done for end-to-end automation of disease detection and management using edge computing.

## 3. Materials and Methods

### 3.1. Dataset

The CXR dataset used in this study is freely available for academic use and can be downloaded from here [5]. It is an evolving dataset, which gets updated every few months. The reason for choosing this dataset is that its large in sample size and is freely available for academic and research purposes. Effective applications begin with data in this era of the latest technology and incredible computational power. During the prevalent COVID-19 situation, organizations concerned about healthcare are emphasizing the collection and storage of different types of data. The data may appear in different forms, such as diagnostic reports, genome sequences, 2D structures, images, biomedical signals, and various features like the patient's age, sex, comorbidities, location, symptoms, etc. The dataset used in this study contains a total of 15,153 X-ray images belonging to three categories. The dataset contains 1,345 viral pneumonia samples (8.87%), 3,616 COVID-19-positive samples (23.87%), and 10,192 normal samples (67.26%).  Figure 1 shows some of the sample CXR images from the dataset. It is evident from Figure 2 that there is a class imbalance.

### 3.2. Hybrid Class Balancing Using Over-sampling and Proportionate Class Weights

Unbalanced datasets are a prevalent problem that will inevitably occur in disease diagnosis data collection. This issue arises when one group of classes has a significant advantage over another. As a result, the machine learning model becomes more biased towards the majority class. It leads to the misclassification of minority groups. In the present case, the dataset has an imbalance of almost the proportion of 1 : 3:8 (viral pneumonia: COVID-19: normal). Here, we apply a two-step process to mitigate the effect of the class imbalance.

#### 3.2.1. Creating New Samples for Minority Classes

New samples are generated for the two new minority classes using the synthetic minority over-sampling technique (SMOTE) as described in [37]. As a result, the new ratio of class samples becomes 1 : 2 : 3. Equisampling the majority and minority classes may lead to overfitting and a lower AUC score. Therefore, selective downsampling of majority class along with SMOTE was suggested by Chawla et al. [37] to mitigate this issue. The majority class is not taken into account when making synthetic examples, which can lead to confusing examples when there is a lot of overlap between the classes. In the current case, the dataset has a class imbalance (1 : 2 : 3), which is corrected in the next stage.

#### 3.2.2. Proportionate Class Weight Assignment

Weighted neural networks or cost-sensitive neural networks are backpropagation algorithms that may be adjusted to weight misclassification mistakes in proportion to the relevance of the class. In datasets with a strongly skewed class distribution, this allows the model to pay more attention to samples from the minority class than the majority class. The majority class's decrease in error is substantially scaled down to very tiny numbers, which may have only a slight or no influence on model weights. We assign class weights of 0.50, 0.33, and 0.17 to further mitigate the effect of class imbalance.

### 3.3. Image Enhancement

To eliminate even a small amount of noise, picture smoothing methods such as Gaussian blurring, bilateral filtering, and others are used. The Gaussian filter is a filter that is commonly used in image processing to smooth out images, reduce noise, and compute derivatives. It is a convolutional filter with Gaussian matrices as the underlying kernel. The reduction of noise from the original input picture is shown in Figure 3. A Gaussian function in two dimensions has the following formula:

(1) $$\begin{array}{c} G\left(a,b\right)=\frac{1}{2\pi \sigma^{2}}e^{-\left(a^{2}+b^{2}/2\sigma^{2}\right)}. \end{array}$$

### 3.4. Data Augmentation

Data augmentation is the strategy of manipulating existing data to create new data objects. Rotating, resizing, cropping, and other techniques can be utilized to augment new image samples from the existing set. It is critical to investigate the process's resilience in preserving the same label after transformation while using data augmentation. Rotations and flips, for example, are usually resilient on detection tests like cat vs. dog, but not on digit identification tasks like 6 vs. 9. In image classification, object recognition, and segmentation, data augmentation may be utilized entirely to train deep learning models.  Table 1 lists the type of data augmentation transformation applied to the dataset. Different data augmentation transformations are shown in Figure 4.

### 3.5. Data Preprocessing

Neural networks learn best from small values. Some simple transformations, conversions, and scaling, collectively known as preprocessing steps, may be helpful. It is a crucial step to making the data fit for a machine learning model. There may be some inadvertent noise and artefacts during the acquisition of data, such as gel application prior to CXR image capture. To achieve a high classification rate, we eliminated noise and objects from the images. We have used data normalization, data elimination, feature extraction, and, eventually, numerical data to convert the string data of the mark.

### 3.6. CNN Hyper-parameter Tuning

The CNN hyper-parameter tuning was also done. On the other hand, CNN hyper-parameter optimization seeks to identify the best range of values for a given dataset before training can begin in a suitable period of time (e.g., the number of epochs). The introduction of residual connections overcomes the degradation problem caused by deep structures while simultaneously shortening the training period. It is capable of obtaining superior results to other CNN designs.

### 3.7. Custom Deep Learning Model Architecture

Transfer learning is a branch of machine learning that aims to transfer data from a source model to a target project by using correlations in outcomes, functions, or models. It may obey a range of distributions, and data annotation does not require a large number of annotations. The simulation model's characteristics and weights will be used to train new models and completely new tasks. The training model's characteristics and weights will be used to train new models and complete new activities in the model. Transfer learning makes it possible to use a previously trained model's experience (features, weights, and so on) to train a newer model and is beneficial in many ways, including getting fewer data points for the new mission. For transfer learning, the Inception-Resnet-V2 architecture with pretrained weights was used. We froze the weights of the starting 100 layers in the custom model. The learned network does not change the parameters of the frozen layers. Many initial layer weights may be frozen to speed up network training and avoid overfitting of the dataset. The ImageNet dataset containing over a million images was used to train the CNN model Inception-ResNet-v2. There are 164 layers in the network that can categorize around 1000 object categories. As a result, the network model is capable of learning rich attribute representations for a variety of images. Multiple-sized convolutional filters and residual connections are merged in the Inception-Resnet block. The motivation for choosing this architecture is based on the experimental results and comparative analysis with other popular deep learning models (presented in Section 6). Inception-ResNet-v2 presents a nice trade-off between model performance (accuracy) and resource requirements. As the model was supposed to work in an edge environment, other resource-extensive, bulky models could not be chosen.  Figure 5 depicts the architecture of the custom model.

Residual connections provide for model shortcuts, allowing this architecture to achieve even higher performance. It allows some simplification of the Inception blocks. This design is a hybrid of Inception and residual blocks that improves performance. To enhance the training outcome, Inception makes better use of computational resources and can extract more features with the same amount of computation. The output of the preceding layer is combined within the network since the calculation of the 5 × 5 convolution kernel is too large. The 1 × 1 convolution is used throughout the Inception module for two reasons: the first is to superimpose further convolutions over receptive fields of the same scale in order to derive richer features from the constellation diagram, and the second is to reduce the measurements and computational cost. The network's 1 × 1 convolution, which comes before the 3 × 3 and 5 × 5 convolutions, is used to reduce dimensionality. Figuring out the optimal hyper-parameter values is an important part in transfer learning models. Finding the right balance between underfitting and overfitting is the goal of this approach. It involves examining the loss and accuracy for indications of underfitting and overfitting in order to strive for the most optimal set of hyper-parameters and then optimizing them.  Table 2 lists various model hyper-parameters and their respective values. These are learning rate (LR), momentum, dropout rate (DR), kernel size (KS), max pooling, initial weight scaling (IWS), and hue shift (HS).

Dense layers use the rectified linear unit (ReLU) activation function that can be mathematically defined using following equation:

(2) $$\begin{array}{c} R\left(z\right)=\max\left(0,Z\right). \end{array}$$

The fully linked layer was replaced with global average pooling, with the exception of the Inception module. This was done to reduce the number of variables. Batch normalization (BN) also forms part of the network at the same time. The BN layer will make each mini-batch constellation map the same as it moves up to a neural network layer, preventing gradients from disappearing.

It is a set of constellations that serves as the training ground for any given constellation. In the backpropagation algorithm, we must also calculate Jacobians. These are simply partial derivations of the norms for the variables *a* and *x*.

(3) $$\begin{array}{c} \frac{\partial \text{Norm}\left(a,\chi \right)}{\partial a}\mathrm{and}\frac{\partial \text{Norm}\left(a,\chi \right)}{\partial \chi }. \end{array}$$

In the network, Adam is used to maximize the network parameter and minimize the loss. When working with large problems with a lot of data or parameters, the method is extremely efficient. It is efficient and requires less memory.

(4) $$\begin{array}{c} \theta_{x}≔\theta_{x-1}-\alpha \cdot \frac{{\hat{m}}_{x}}{{\sqrt{v}}_{x}+\varepsilon }. \end{array}$$

Here, *α* ∈ *R* and $\theta ,{\hat{m}}_{t},{\hat{v}}_{t},\epsilon \in R^{n}$ for some *n*.

To avoid overfitting, dropout may be helpful as a regularization technique. For the most part, dropout refers to the fact that during training, with a certain probability *p*, a neuron of the neural network is turned off. The equation for dropout is given for probability *p*_i_ (1 ≤ *i*<=*t*) below:

(5) $$\begin{array}{c} E_{R}=\frac{1}{2}{\left(x-\sum_{i=1}^{t}p_{i}w_{i}I_{i}\right)}^{2}+\sum_{i=1}^{t}p_{i}\left(1-p_{i}\right)w_{i}^{2}I_{i}^{2}a. \end{array}$$

Figure 6 depicts the major steps of the proposed training process on the dataset.

### 3.8. Edge Computing-Enabled Prediction System

There are many IoT and edge deployment options available in the market from the leading players such as Google, Amazon, Microsoft, and IBM. A comparison of some of these solutions and architectures has been provided in [38]. The system was deployed on Amazon IoT Core (AIC) using the MQTT protocol and an Amazon S3 bucket was used for data storage. MQTT is a simple subscribe/publish model-based communication protocol. The alternatives and contenders to MQTT are Google Cloud Messaging, RabbitMQ, XMPP, and Kafka. Due to its low resource consumption and lightweight characteristics, it is extensively used in edge environments for communication and message passing [39]. In AIC, for data storage, there are a couple of options available. DynamoDB is a very widely used database option. However, it can only send data up to 64 KB, which is not suitable for sending X-ray images. That is why we chose Amazon S3, which can accommodate as much as 5 TB of data. Furthermore, it becomes very convenient to access these data for a web interface display.

An edge computing-enabled system has been implemented to make the disease classification process happen in a seamless way.  Figure 7 depicts the layered edge architecture of the system. It has been divided into four layers, namely the physical layer, the edge computing layer, the network layer, and the application layer. The bottommost layer is the physical layer that has an array of CXR acquisition machines (*M*_1_, *M*_2_,..., *M*_*n*_). The data captured by the physical layer move to the next layer, that is, the edge layer. Most of the analytical processing on image data takes place here. The edge layer contains an array of edge nodes (*N*_1_, *N*_2_,..., *N*_*n*_). A typical edge node is a Raspberry Pi 4 setup with 8 GB of RAM and has wireless network connectivity. Every device we want to connect to in the AIC ecosystem is a “thing.” We need to register the “things” before being able to communicate with them. The MQTT message protocol is used for this purpose. The authentication code needs to be copied on each of the devices. Bulk device regionalization is also possible to connect more than one device (or thing). A certificate-based security mechanism is followed. We need to download the public key, private key, the regular certificate, and the root CA for AWS that supports SSL to securely connect to AWS. All these documents need to be pushed to the edge nodes, and that can be done with the help of a file transfer protocol (FTP) client. We use FileZilla for this purpose.

The custom deep learning model trained in Section 3.7 is run on each edge node for image classification. CXR images are registered and mapped with a unique patient identification number (PID) and can be managed from the cloud application. The edge layer is further connected to the network layer in order to have access to the cloud. All the analytics and disease diagnosis data are pushed to the cloud server. The topmost layer in the architecture is the application layer that runs many useful functions, such as report generation, notification management, outbreak prediction, etc. This layer can enable role-based access to these services.

## 4. Comparison with Other Deep Learning Models

### 4.1. VGG19

VGG19 is a deep learning architecture model that was previously trained to detect image representations on a large-scale image dataset also known as ImageNet. The model achieves 92.7 percent top-5 evaluation accuracy in ImageNet. When compared to other more complex models, it achieves competitive classification accuracy. It is linked to the fact that it has a strong structure. There are different sets of convolution layers, each having 64 filters, 128 filters, 256 filters, and 512 filters in a particular order. Each series of convolution layers contains max pooling layers. 2 × 2 filters with a stride of 2 are used in max pooling layers (pixels). The output of the final pooling layer is flattened and subsequently fed to a fully connected layer with 4096 neurons that is used for classification. This output is further received as input to a fully connected layer having 4096 neurons. What this layer produces is fed to another fully connected layer having 1000 neurons. There are other subsequent layers with ReLU activation and finally the softmax layer.

### 4.2. ResNet50

ResNet is the abbreviation for residual networks, a form of neural network. It is a 50-layer convolutional neural network (CNN). ResNet's core idea is to present a so-called “character alternative way association” that bypasses at least one layer. There are 23,587,712 parameters in the standard ResNet50 model, which can classify images into 1,000 object categories. It consists of a convolutional kernel of size 7 × 7 along with 64 individual kernels, both with a size and stride of 2, and max pooling with the same stride scale as the kernels.

### 4.3. MobileNetV2

MobileNetV2 contains two blocks, namely the one-stride residual and the two-stride residual block. Both types of blocks have three layers. The first layer happens to be a 1 × 1 convolution with an improved activation called ReLU6. The depthwise convolution is the last step. Another 1 × 1 convolution without nonlinearity is used in the third layer. The inner layer encodes the model's ability to learn from lower level features (like pixels) to higher level descriptors. Further, the bottlenecks encode the model's ability to modify from lower level descriptors to higher level descriptors.

### 4.4. CNN (Convolutional Neural Network)

In CNN, six convolutional layers with channel sizes of 96, 96, 128, 128, 128, and 128 are used. The 3 × 3 filter size, 1 stride length, and ReLU activation functions are used in each of these layers. There were three max pooling layers overall, each with a size of 2 × 2 and a stride of 2. A 50% dropout rate was utilized after each pooling layer, and in the fully linked layers, an L2 regularization was used to counteract overfitting (with a hyper-parameter of 0.0005). Also included are three completely linked layers with sizes of 1024, 512, and 10, with ReLU activation on the first two and softmax on the third.

## 5. Comparison with Machine Learning Models

### 5.1. Local Binary Pattern (LBP)-Based Support Vector Machine (SVM) Classifier

SVM was chosen because it employs the kernel method to transform low-dimensional input space to high-dimensional input space, thereby converting a nonseparable representation into a separable one [40]. Unlike the convolution-based models (ConvNets), where feature extraction is part of an end-to-end process [41], SVM relies on the need for a feature extraction step. The SVM classifier uses a hyperplane to linearly separate the data using the linear kernel. Parallel hyperplanes divide each data class, ensuring that the distance between them is as vast as feasible. As, we are dealing with the very high-priority circumstance of identifying COVID-19, we are searching for a narrower margin hyperplane to categorize the infected classes more correctly with fewer miss-predictions. The SVM is trained using LBP features from both folded and unfolded pictures. It converts a greyscale picture to a matrix of integer values at the pixel level. The original picture is described by this label matrix. It calculates the texture's local representation. It is a visual description that is utilized in computer vision to categorize items. The LBP for a given pixel neighbourhood (*gp*_*x*_,*gp*_*y*_) coming from sampling distribution of *gp* and centered around *gc* can be calculated using the following equation:

(6) $$\begin{array}{c} LBP\left(gp_{x},gp_{y}\right)=\sum_{p=0}^{P-1}S\left(gp-gc\right)\times 2^{p}. \end{array}$$

The function *S*(*k*) is a binary output function that returns value 1 when *k* ≥ 0, and it returns value 0 for all negative values. This binary output is cumulatively multiplied with the powers of 2 and summed-up that way.

### 5.2. Histogram of Oriented Gradient (HOG)-Based Decision Tree (DT) Classifier

To generate decision trees, a recursive partition approach is utilized, in which data points are split at each node based on the split criterion set. The path from a root node to a leaf is a rule that is used for prediction. An ensemble of classifiers is made up of several classifiers. The members of the classifiers all get together to make the final decision. An ensemble performs better than the sum of its parts when its individual members are accurate and diversified. Decision tree ensembles are very resistant to perimeter selection and outperform other methods. In the trials, many decision trees based on ensembles are used. The HOG descriptor is concerned with the structure or shape of an item.

The HOG feature descriptor counts the number of occurrences of a gradient orientation in a certain section of an image. HOG may also be used to indicate the edge direction. This is achieved by removing the edge. This is accomplished by extracting the edge gradient *g* and orientation *θ* with the following simple formulae:

(7) $$\begin{array}{c} g=\sqrt{g_{x}^{2}+g_{y}^{2}},\\ \theta =\arctan\frac{g_{y}}{g_{x}}. \end{array}$$

## 6. Results and Discussion

### 6.1. Description of Tools and Experimental Setup Used

The deep learning model training was performed on a workstation with a quad-core processor (Ryzen 7), an NVIDIA Geforce GTX 6 GB GPU, 16 GB of RAM, and the Windows 10 operating system. The networks trained over 100 epochs, with an early stopping point set at a validation loss. Patience was assigned a value of 10. Python's deep learning library Keras with Tensorflow as backend, sklearn, seaborn, matplotlib, and other libraries were used for model creation, training, performance evaluation, and visualization tasks. For feature extraction from the images, MATLAB R2021b version with image processing toolbox was used.

### 6.2. Experimental Results

All of the models were trained for 100 epochs with early stop callback criteria (patience = 20 epochs). We found the Adam optimizer with a learning rate of 0.0001 to be converging faster for our problem. For all three models, the same optimizer is used, and the models are then saved as h5 files.  Figure 8 depicts the plots obtained during training and testing of different models. The loss and accuracy graphs for the custom model are shown in part (A) of Figure 8, while the plots for VGG19, ResNet50, and MobileNetV2 are shown in the (B), (C), and (D) parts, respectively.

The different accuracy metrics for the bespoke approach are shown in Table 3. Precision, recall, and an *F*1 score are all included. The harmonic weighted average of accuracy and recall is the F1 score that takes into account the false positives and false negatives and transmits the delicate balance between accuracy and recall.

(8) $$\begin{array}{c} F1\;\mathrm{Score=}\frac{\mathrm{2x}\left(\mathrm{Precision}\;x\;\mathrm{Recall}\right)}{\left(\mathrm{Precision+Recall}\right)}. \end{array}$$

### 6.3. Mean Accuracies of Different ML Classifiers

Figure 9 shows a plot of the mean accuracies of several ML classifiers. The image depicts the accuracy values for various feature combinations, and as can be observed, the linear regression line for all classifiers increases as the number of features increases.

### 6.4. ROC Curve and Confusion Matrix

Figure 10 shows the ROC curves for the classification of COVID-19, normal, and viral pneumonia. The connection between the false-positive rate (FPR) and the true-positive rate (TPR) is depicted by the receiver operating characteristic (ROC) curve. A depiction of TPR (*y*-axis) and FPR (*x*-axis) is known as a ROC curve (*x*-axis). The TPR and FPR can be calculated with the following formulae :

(9) $$\begin{array}{c} \mathrm{TPR=}\frac{\mathrm{TP}}{\mathrm{TP+FN}},\\ \mathrm{FPR=}\frac{\mathrm{FP}}{\mathrm{FP+TN}}. \end{array}$$

The curve indicates the performance of the deep learning model. We can observe the values of each individual class. The area under the ROC curve (AUC) was calculated to be 99.8%.

Figure 11 depicts the confusion matrix. A confusion matrix is a tabular representation that explains how well a classification model performs. It is an *n* × *n* matrix, with “*n*” indicating the number of classes. In a confusion matrix that compares model class predictions with actual class predictions, type II errors, also known as false negatives, occur in the second quadrant, whereas type I errors (false positives) occur in the third quadrant.

### 6.5. Effect of Data Augmentation on Accuracy Values

The impact of data augmentation on performance measures is shown in Tables 3and 4. As can be seen from the table, data augmentation improves the model's performance since the number of training samples increases without affecting the ratio of picture classes. The loss value is calculated using the categorical cross-entropy function. Models with data augmentation have lower loss values since the real classes are fairly similar to the desired classes.

The Keras deep learning framework's image data generator class is utilized to supplement training samples in this case. When the number of epochs is large, the number of training samples created by the data augmentation approach is quite high when compared to training samples without data augmentation. When data augmentation is used, distinct sets of training samples are created for each epoch. When data augmentation is not used, the same set of training samples is used for each epoch.

### 6.6. Limitations of the Study

When compared to other ML, DL, and TL methods, the proposed technique has produced significantly better results. It is also suitable for use in edge computing environments, as previously mentioned. However, there is still room for further research and improvement in this area in the future. By increasing the number of samples used for training, the proposed method can be made even more effective. Furthermore, a greater number of classes of CXR diseases can be added to make the tool more useful in its current form. Because of the limited availability of data and restrictions on commercial use, it was not feasible to implement in a commercial setting. These difficulties may be taken into consideration, and they may serve as a source of motivation for future research.

## 7. Conclusion

CXR imaging is a commonly used tool to diagnose various diseases, including COVID-19. Due to an acute shortage of qualified radiologists and in order to assist them in their task of disease detection, an edge computing-based system is proposed in this article. To classify diseases in an openly available CXR image dataset, a variety of machine learning (ML), deep learning (DL), and transfer learning (TL) approaches were evaluated in this study. There lies a class imbalance in dataset. It was tackled with a combination of the synthetic minority over-sampling technique (SMOTE) and weighted class balancing is used. The best accuracy comes from a hybrid Inception-ResNet-v2 transfer learning model. Data augmentation and image enhancement help in improving the accuracy of disease classification task. The proposed technique has a 98.66 percent average accuracy. Other TL models such as SqueezeNet, VGG19, ResNet50, and MobileNetV2 have accuracy of 97.33 percent, 91.66 percent, 90.33 percent, and 76.00 percent, respectively. Furthermore, a DL model that was trained from the scratch has an accuracy of 92.43 percent. Support vector machine with local binary pattern (SVM + LBP) and decision tree with histogram of oriented gradients (DT + HOG) are two feature-based ML classification techniques that have accuracy of 87.98 percent and 86.87 percent, respectively. The model is used in an edge environment with Amazon IoT Core to automate disease detection in CXR images in three categories: pneumonia, COVID-19, and normal. The proposed system is good to be used as an assistive tool for the automated screening tool for COVID-19 and viral pneumonia [41].

## Figures and Tables

**Figure 1:** Sample X-ray images from the dataset.

**Figure 2:** Label count of the classes.

**Figure 3:** Removing noise from the input image.

**Figure 4:** Data augmentation during training: (a) original, (b) rotated, (c) zoomed, (d) vertically shifted, and (e) horizontally shifted.

**Figure 5:** The architecture of the custom model.

**Figure 6:** Schematic flow diagram of the proposed system.

**Figure 7:** Layered architecture of the edge enabled system.

**Figure 8:** Accuracy and loss of comparison of (a) proposed custom model, (b) VGG19, (c) ResNet 50, and (d) MobileNetV2.

**Figure 9:** Mean accuracies of CNN and two different ML (SVM and decision tree)-based classifiers.

**Figure 10:** ROC curve.

**Figure 11:** Confusion matrix of the custom model.

**Table 1:** Parametric values used for data augmentation.

Parameter	Value
Channel shift range	10
Fill mode	Nearest
Height shift range	0.4
Horizontal flip	TRUE
Rotation range	5
Shear range	0.25
Width shift range	0.3
Zoom range	0.25

**Table 2:** Model hyper-parameters and their values.

Hyper-parameter	Range
DR	[0, 0.6]
HS	[0, 40]
IWS	[0, 2.0]
KS	{1, 3}
LR	[0.0001, 0.001]
Max pooling	{True, false}
Momentum	[0.68, 0.99]

**Table 3:** Performance comparison of different models.

Model	Class	Accuracy	Precision	Recall	*F*1-SCORE
*Custom*	COVID-19 class	0.99	0.99	0.99	0.99
	Viral pneumonia class	0.99	0.99	0.99	0.99
	Normal class	0.98	0.99	0.98	0.98

*VGG19*	COVID-19 class	0.98	0.98	0.99	0.98
	Viral pneumonia class	0.89	0.90	0.89	0.89
	Normal class	0.88	0.88	0.88	0.88

*ResNet50*	COVID-19 class	0.87	0.87	0.87	0.88
	Viral pneumonia class	0.92	0.93	0.92	0.92
	Normal class	0.92	0.93	0.92	0.92

*MobileNetV2*	COVID-19 class	0.79	0.79	0.80	0.79
	Viral pneumonia class	0.75	0.75	0.75	0.75
	Normal class	0.74	0.74	0.76	0.75

*SqueezeNet*	COVID-19 class	0.98	0.98	0.98	0.98
	Viral pneumonia class	0.96	0.96	0.98	0.97
	Normal class	0.98	0.98	0.98	0.98

**Table 4:** Effect of data augmentation on performance.

Metric	Proposed model	
	With augmented data (%)	Without augmented data (%)
Training accuracy	99.5	92
Validation accuracy	98.5	91
Test accuracy	99.6	91

## Data Availability

The CXR dataset can be accessed from the source mentioned in reference [5].
